RETRACTED

# Analysis of the Effect of Artificial Intelligence on Role Cognition in the Education System

**DOI:** 10.1155/2022/1781662

**Published:** 2022-05-30

**Authors:** Jianjian Zhu, Chuming Ren

**Affiliations:** ^1^Department of Public Administration, Xi'an University of Finance and Economics, Xi'an, Shaanxi 710016, China; ^2^International College, Krirk University, Bangkok, Thailand

## Abstract

Taking the entire education system in Taiyuan City, Shanxi Province, Central China, as an example, this paper uses the questionnaire survey method to analyze the effect of artificial intelligence (AI) on role cognition in the education system. The education system targeted by this questionnaire survey involves 8 categories: preschool education, primary education, secondary education, higher education, adult education, computer network education, enterprise education, and social education; the respondents include 368 teachers, 402 students or learners, 118 school managers, and 124 family members of students or learners in all above education categories. The questionnaire design has a total of 34 question classified into 6 role cognition items, with a 5-level score; a total of 1012 questionnaires were distributed, and 978 were recovered with a recovery rate of 96.64%, in which 957 were valid questionnaires with an effective rate of 97.85%. The study results show that the learning of AI-assisted courses is strongly dependent on course role cognition, and the construction of role cognition is related to the understanding of course content, teaching methods, and activity methods. Therefore, the effect of AI on role cognition in the education system needs to be systematically analyzed from the aspects of function realization form, resource presentation method, supporting hardware form, teacher-student interaction method, and representation method of works. As connecters, teacher's role cognition is limited by the degree of understanding learners, the amount of resources, and data processing capabilities, but the advantage is that they can flexibly monitor and adjust. AI technology is flexible and diverse, it functions in learning and teaching activities in a variety of ways, and there is no agreement on the terminology to describe its role in role recognition. The results of this paper provide a reference for further researches on the effect of AI on role cognition in the education system.

## 1. Introduction

Artificial intelligence (AI) capable of autonomous perception, understanding, prediction, and action is an unprecedented powerful learning technology, which enhances the flexibility and adaptability of computers as interactive subjects in the process of teaching and learning. In the context of promoting the research and practice of AI education on a large scale, it is very necessary to systematically sort out the microscopic mode of action and role cognition of AI in supporting learning and teaching [1]. In this process, the cognitive analysis of the teaching role of AI will be a very effective entry point. At the first level, AI systems are designed to be used in a formal school setting, where teachers use computer systems to present knowledge to students. In the second level, the computer system will focus on the learning of the students and help the students to learn through intelligent machines but only at the most superficial level [2]. In the third-level stage, the intelligent system gradually exerts its ability to perceive, plan, reason, and make decisions to help teachers to complete teaching. The role in the sense of social psychology refers to the position an individual occupies in a certain social relationship and its prescribed behavior pattern [3]. The role of teachers is to promote people's growth, which includes two dimensions: teaching and educating people. In the fields of knowledge transfer, knowledge organization, and knowledge management, more and more jobs will be replaced by AI. For a computer system, behavior is equivalent to the function it provides, and role is a collection of specific functions [4].

RETRACTED

The arrival of the era of AI has had a huge impact on role cognition in the traditional education system, requiring teachers to establish a new concept of talents, teachers and students, and teaching concepts, and reunderstand the role of teachers. Although each scholar has different views on role cognition, they all share a common view that role cognition is the early stage of the role development process [5]. For teachers, before changing their roles, they must first understand the roles they should play and clarify their functions and obligations. Therefore, role cognition is the premise of role identification and a prerequisite for role transformation [6]. The awareness and ability of AI education application of institutions and individuals vary greatly, and they are generally low. As a connecter, teachers are limited by the degree of understanding learners, the amount of resources, and data processing capabilities, but the advantage is that they can flexibly monitor and adjust. Teachers not only assume the role of knowledge imparting but also need to have good intellectual literacy and cultivate students' core literacy and moral sentiment. Students are no longer passive receivers of knowledge and need to be transformed into knowledge seekers and active acquirers [7]. Under the guidance of teachers and the assistance of AI, they need to acquire knowledge, participate in practice, and improve their innovation capabilities through human-machine collaboration methods to achieve personalized learning [8].

RETRACTED

Taking the entire education system in Taiyuan City, Shanxi Province, Central China, as an example, this paper uses the questionnaire survey method to analyze the effect of AI on role cognition in the education system. The education system targeted by this questionnaire survey involves 8 categories: preschool education, primary education, secondary education, higher education, adult education, computer network education, enterprise education, and social education; the respondents include 368 teachers, 402 students or learners, 118 school managers, and 124 family members of students or learners in all above education categories. Taking secondary education as an example, the sample selection first randomly selects a class of five grade students in each school and then selects students with odd student numbers in each class as the survey object. For the convenience of the survey and to ensure the randomness of the sample, the parents or relatives of the selected student sample are taken as the family sample. The teacher sample was identified as qualified and full-time teachers, excluding principals, deans, and other administrators and service personnel. The detailed chapter arrangement is as follows: Section 2 introduces research methods and data acquisition.  Section 3 is survey result analysis.  Section 4 is discussion.  Section 5 is conclusion.

## 2. Research Methods and Data Acquisition

### 2.1. Questionnaire Design

Using the method of questionnaire survey, this study takes the entire education system of Taiyuan City, Shanxi Province in Central China as an example to explore the effect of AI on role cognition in the education system. The education system targeted by the questionnaire involves school education system, computer network education system, enterprise education system, and social education system; the school education system also includes preschool education, primary education, secondary education, higher education, and adult education. The objects of the questionnaire design include teachers, students, administrators, and family members of various education categories. The questionnaire sorted out a total of 64 descriptions of the role cognition of various objects in various educational systems and then further sorted out the descriptions into 34 questions. Finally, according to literature materials, these 34 questions were classified as 6 role recognition items. The questionnaire uses a 5-level score, and the subjects are asked to make a choice of “extremely important,” “very important,” “relatively important,” “not very important,” and “not important” for each question listed in the above order and make a 5-point rating of 5-1 (Table 1).

RETRACTED

### 2.2. Questionnaire Structure

The questionnaire of this study includes three parts: basic information, investigation themes, supplementary questions, and open-ended questions. The investigation subject part consists of 34 questions and is classified into 6 role cognition items: morality and discipline, knowledge and professionalism, activities and communication, guidance and consultation, research and practice, and goals and feedback. The thematic parts of the questionnaires used in this study for teachers, students, administrators, and families are consistent with each other and aim to understand the perceptions and attitudes of various object roles in various education systems with the possibility of side-by-side comparisons. At the end of each questionnaire, supplementary items of self-made questions are designed, such as “please write the questions that you think are important but not listed in the question, and give the corresponding score.” An open-ended question was also designed at the end of each questionnaire: “What other suggestions do you have,” aiming to further obtain more materials to have a more comprehensive understanding of the effect of AI in the effect of AI in the education system.

### 2.3. Sample Selection

The selection of the questionnaire survey sample adopts the combination of purposeful sampling and random sampling. A total of 5 units in each of the preschool education, primary education, secondary education, high education, adult education, network education, enterprise education, and social education in Taiyuan City, Shanxi Province, were selected, including 368 teachers, 402 students or learners, 118 school managers, and 124 family members of students or learners. The detailed sampling distribution of each system is shown in Table 2. Taking secondary education as an example, the sample selection first randomly selects a class of five grade students in each school and then selects students with odd student numbers in each class as the survey object. For the convenience of the survey and to ensure the randomness of the sample, the parents or relatives of the selected student sample are taken as the family sample. The teacher sample was identified as qualified and full-time teachers, excluding principals, deans, and other administrators and service personnel.

### 2.4. Questionnaire Distribution and Recovery

Teacher questionnaires were distributed and recovered with the assistance of the educational affairs department of the surveyed units; a total of 368 questionnaires were distributed, and 348 were recovered with a recovery rate of 94.57%, in which 343 were valid questionnaires with an effective rate of 98.56%. The student questionnaires were distributed and recovered by a combination of online and offline methods; a total of 402 questionnaires were distributed, and 399 questionnaires were recovered with a recovery rate of 99.25%, in which 393 were valid questionnaires with an effective rate of 98.50%. The school manager was distributed and recovered with the assistance of management department of the surveyed unit; a total of 118 questionnaires were distributed, and 118 were recovered with a recovery rate of 100%, in which 117 were valid questionnaires with an effective rate of 99.15%. The family questionnaires were distributed and recovered by means of online links; a total of 124 questionnaires were distributed, and 113 were recovered with a recovery rate of 91.13%, in which 104 were valid questionnaires with an effective rate of 92.04% (Table 3).

RETRACTED

### 2.5. Questionnaire Data Statistics

Statistical analysis was carried out on 34 questions in the main part of the survey, text analysis was used for self-made questions and open-ended questions, and they were classified as qualitative analysis. SPSS 19.0 statistical software was used for statistical processing, the input data were analyzed, and the measurement data were expressed as mean ± standard deviation. The *t*-test and one-way analysis of variance were used to analyze the effect of AI on role cognition in the education system.

## 3. Results and Analyses

### 3.1. Effect of AI on Role Cognition in Different Education Categories

From a psychological point of view, role cognition is the foundation, and role behavior is the foothold. Therefore, this study discusses in the order of role cognition, role emotion, and role behavior and regards role identification as a structure that integrates knowledge, emotion, and behavior. The learning of AI courses is strongly dependent on course role cognition, and the construction of role cognition is related to the understanding of course content, teaching methods, and activities. The form of function realization, the way of resource presentation, the form of supporting hardware, the way of interaction between teachers and students, and the way of representation of works are systematically analyzed. The design and practice of the cognition of the learning roles in the course support are highly consistent with the educational concept and value cognition of the AI course. Most of the supporting role cognition used in the current AI course teaching is based on code programming or graphical programming, and some schools have participated in the development of some learning role cognition [9]. Most of these role cognitions provide support in terms of technical experience, user innovation, code or graphical programming, virtual or materialized presentation, and related kits, and a few also provide certain teaching resources or knowledge sharing inside and outside of role cognition. Most of them do not provide teaching support services such as real-time interaction between teachers and students. The effects of AI on role cognition of teachers or couches, students or learners, school managers, and family members in different education categories are shown in Figure 1.

RETRACTED

With the support of AI technology, respecting the individual characteristics of learners and providing personalized guidance for learners is about to become a reality. Based on the learner's personal information, cognitive characteristics, learning records, location information, media social information, and other databases, the AI program can self-learn and build a learner model and continuously adjust and optimize the model parameters based on the expanded and updated data set, thereby realizing the push of personalized resources, learning paths, and learning services. The clearer the individual's cognition of the theoretical positioning of the role, the more successful the role plays; otherwise, it may lead to the failure of the role. Role cognition is also the premise and foundation of role behavior. There is still a big difference between face-to-face communication and face-to-face interaction between people. For the learning of students in school, it is necessary to respect the knowledge structure of the course, take into account the students' learning interests, and discover hidden laws based on data such as learning content, teacher suggestions, students' interests, and learning behaviors, so as to build an effective learning support model [10].

The analysis of the effect of AI in the education system is characterized by active intervention in the learning process of students according to the cognitive characteristics of different students on the basis of data analysis, so as to optimize the learning process and scientifically evaluate learning effectiveness. The adaptive learning system based on cognitive level ability can apply the model to guide, intervene, optimize the learning process, and make scientific evaluation, which can be regarded as a system with real intelligent and adaptive functions. The application of AI technology in the establishment of students' personalized learning space, optimization of personal learning process, and improvement of learning efficiency can be expected, and its value is relatively easy to judge. The effect of AI is far lower than the role that students can play in the process of propositional knowledge learning. But in fact, on the one hand, the data processed by the perception layer is quite scarce, which greatly restricts the possibility of perceiving students' knowledge level and learning status through AI; therefore, it is still difficult to produce a truly intelligent and adaptive system.

RETRACTED

### 3.2. Effect of AI on Role Cognition of Different Research Objects

In role identity theory, scholars believe that role identity includes multiple dimensions, such as role cognition, role emotion, and role behavior. The feelings expressed by the individual's evaluation of the role cognition and the role affection are affected by the individual's experience of the role played and the environment in which the role is located. The combination of AI technology and education and teaching system has greatly improved the interaction between teachers and students in classroom teaching and the uniqueness of the education model [11]. The popularization of AI in school teaching will objectively force teachers to rethink and clarify their majors by the problem of role positioning. Teachers should also guide students of all ages to form values and rational thinking that coexist harmoniously with AI in learning and life, so that they can fully understand AI as a technology and tool even if it thrives. One of the main characteristics of AI is that it can learn actively, it can consciously capture practical and demand information in the network for users, and it is more efficient than human data query and sorting (Figure 2). For the question of correctness, teachers and students can also communicate in real time through the system during the teaching process, so as to discover the gaps and deficiencies in learning in time, which is conducive to the realization of personalized learning methods and enhances the interaction between teachers and students.

According to the different forms of existence, roles can be divided into three levels: expected roles, comprehension roles, and practical roles. An expected role is a set of ideal behavioral norms and action patterns set by a society or an organization for a specific social role; so, it is sometimes called an ideal role. The comprehension role is the behavioral norm and action mode that the individual understands, recognizes, and internalizes to the level of concept and consciousness. Practical roles are the practical behaviors and results that individuals show in the process of playing roles and performing normative duties according to their understanding of roles [12]. When an individual's practical role does not match his comprehension role, or when the role expectations raised by the multiple roles that an individual needs to play at the same time are inconsistent, there may be distress, confusion, contradiction, tension, depression, and other negative psychological emotions. Role conflicts in the education system include interrole conflicts and intrarole conflicts. Interrole conflict mainly refers to the bad psychological emotions caused by an individual playing two or more roles with different expectations and requirements at the same time. Intrarole conflict refers to psychological conflicts caused by people outside the role-player who have different cognitions and expectations for the same role or the role-player's own confusion and blurred understanding of role expectations.

RETRACTED

Artificial intelligence has a positive and significant impact on both the cognitive and noncognitive levels of roles in the education system, and the effect at the cognitive level is higher than that at the noncognitive level. At the same time, AI has a positive effect on students' creative thinking ability, problem-solving ability, and academic performance. It further shows that AI has great potential in cultivating students' multiple abilities. Making full use of the advantages of AI's teaching aids to design courses will bring about the improvement of students' cognitive ability in different dimensions. AI has positive effects in different school stages, and the effect is the best in primary schools. The analysis results show that AI has positive and significant effects in elementary school, junior high school, high school, and university, and the effect is the best in elementary school, achieving a highly significant effect [13]. Under the premise of accurately comprehending the correct meaning of various role expectations, they examine and check whether they have the corresponding knowledge, technology, and ability training according to the content of role expectations and then make up and consolidate them in a targeted manner. Only by improving the level of role comprehension can lay the foundation for role practice, and only by improving the level of role competency can the gap between the actual role and the expected role be narrowed, thereby weakening the adverse effects of role conflict.

## 4. Discussions

### 4.1. Correlation Analysis of AI and Role Cognition in the Education System

Artificial intelligence is sometimes unable to achieve detailed and emotional education; so, teachers should be confident in their status and role as educators. The effect of AI in the education system can be analyzed through the three core driving forces of big data, cloud computing, and deep learning to track and record the learning process of learners, pay more attention to the behavior and emotional changes of students, and analyze them according to AI. The data of intelligent statistics further analyzes the law of students' emotional changes and the incentives that cause emotional changes. The role cognition in the education system can take targeted and effective positive intervention methods to guide students to adjust and control their emotions, which is conducive to the sense of belonging, security, and identity of the role, thus producing a positive emotional experience. As shown in Figure 3, teachers should carefully observe students' emotions, the degree of motor development, and the level of social development. Teachers make statistics on students' daily behaviors and life trajectories through big data, which is more convenient and effective to provide scientific and effective basis for teachers to evaluate students' behaviors. The AI evaluates and identifies the level and degree of students' learning and development and proposes improvement suggestions or measures to carry out targeted and appropriate guidance [14].

RETRACTED

Teachers should have the courage to face reality, constantly enrich their literacy, and do a good job in information-based teaching and handle the cooperation and distribution relationship between teachers and AI. Facing the ever-developing AI technology environment, teachers should do a good job in coping with implementation, accurately positioning their own work, rationally distributing workload, and realizing human-machine symbiosis. Teachers should pass on moral emotions and logical innovative thinking to students, so that knowledge is always passed on in emotions, which is a human characteristic that cannot be replaced by AI. The natural learning environment includes teaching objects and public facilities in the real teaching environment. Teachers should reflect the subjectivity of students in environmental design [15]. All environmental design is carried out around students' learning. The arrangement of seats should help teachers and students and their interactions. Teachers show students a wealth of learning resources through electronic devices, and teachers and students achieve a tacit understanding of teaching and learning through the physical environment. In teaching, teachers should guide students to learn self-inspection and self-assess their own performance to find their own shortcomings. Teachers should also use various data collected by AI technology to design different learning plans to meet students' individual learning needs. Teachers' guidance to students' learning must conform to the physical and mental characteristics of students and promote students' autonomous cognition and ability construction and the formation of ideological awareness.

RETRACTED

AI technology may already play the role of teachers in the education system and perform their knowledge imparting responsibilities, which will also lead to the gradual weakening of teachers' identity and status as knowledge imparters. The knowledge level of students is no longer the only criterion for measuring the quality of school education. The so-called good school is a school where teachers can give full play to their own advantages and values and can cultivate students' information literacy, coordination, and cooperation with AI: a school for innovative thinking and creativity to better adapt to the future society. According to this, some scholars have asserted that the work form of teachers in the future will not focus on teaching, and their responsibility will no longer be knowledge instillation [16]. The effect of AI on role cognition in the education system further improves the accuracy and efficiency of retrieval. As a comprehensive science and technology, AI itself conforms to the characteristics of a variety of professional skills. The education system can make use of this characteristic or expand on the original basis to meet the needs of students' own learning needs. After all, it cannot replace human learning and innovation. This is the subjective condition for students to form a correct learning attitude and motivation to further enhance their independent learning ability and creativity.

### 4.2. Mechanism by which AI Affects Role Cognition in the Education System

Role cognition is the premise and prerequisite of role transformation; role cognition is the key factor affecting role identity. The social role theory holds that individual role-playing is mainly affected by two factors: internal and external factors. The external factor is people's social expectations for the role, and the internal factor is the individual's role cognition. This kind of personalization will increasingly show the characteristics of objectivity and quantification. In a certain social situation, the social function of the role is displayed through the behavior of the subject, which is a collection of its behavior. Teachers can only meet expectations in behavior if they know what role they should assume in their ideological understanding. Teaching role cognition is a general metaphor for the role or way in which a computer system supported by AI technology plays a role in promoting learners' learning process (Figure 4). In the education system, it has not been long before intelligent technology can be used at low cost and on a large scale. Teachers should guide students to gradually form independent self in the process of exploring and understanding themselves based on the concept of taking students as the center; so, it is an important prerequisite to promote the development of their individual values and rationality in future society. AI technology is flexible and diverse, it functions in various ways in learning and teaching activities, and there is no consensus on the terminology to describe its role [17].

RETRACTED

Table 4 shows the rating results of effects of AI on different role recognition descriptions in in the education system in Taiyuan City. The effect of AI in the education system can be analyzed from the aspects of learning new knowledge, review and consolidation, and testing, but the more reliable method is testing. The test scores are the basis for the final determination of mastery. When the mastery of a concept is determined, the learning of other concepts related to this concept will be affected. Because at the beginning of the project research, it was assumed that there is a logical relationship within the learning materials, and the cognition of each role is related to each other. The degree of concept mastery, the learner's role cognition level, and the logical relationship between concepts jointly determine the difficulty level and complexity of new knowledge pushed by AI for learning. Role cognition in the education system is identified by the load change curve of AI, where the maximum cognitive load is the maximum load level that the learner can handle. The measurement parameters of role cognition in the educational system are expressed in response time. From experimental data and psychological theory, it can be concluded that although each person's student model parameters have the same dimensions, due to each person's different knowledge backgrounds, learning styles, etc., different learners will invest in a certain knowledge point. Therefore, it is necessary to include the cognitive load characteristics of learners.

In the era of AI, in the process of promoting intelligent education, teachers and students are prone to risks in the transformation of teaching roles. For teachers, role change is a change in knowledge structure, teaching methods, and thinking concepts. In addition, through the accumulation of learners' learning data on a regular basis, targeted learning process analysis is carried out, and the weak links of students' learning are more clearly and intuitively understood through big data. However, in the face of the advanced AI technology in the future, some teachers may worry that they will be replaced, or they may not be confident that they can master intelligent technology well. There are also some teachers who may overtrust AI, which leads to the decline of their own abilities and gradually loses their own unique reflection on teaching [18]. For students, role change means changing the concept of learning and the way of learning. Students are no longer passive receivers of knowledge and need to be transformed into knowledge seekers and active acquirers. Under the guidance of teachers and the assistance of AI, they need to acquire knowledge, participate in practice, and improve their innovation capabilities through human-machine collaboration methods to achieve personalized learning.

RETRACTED

### 4.3. Factor Analysis of AI Acting on Role Cognition in the Education System

Since the knowledge organization and reasoning process in the expert system is a simulation of the way of thinking of human experts, the organization of the knowledge base and the systematic reasoning process can better reflect the thinking process of role cognition in the education system. In the process of building a knowledge base, role cognition needs to conceptualize, formalize, and organize the fragmented and unformed knowledge. As shown in Figure 5, the process of building a knowledge base can not only reflect the learning process of role cognition but also help the role cognition to think deeply about knowledge and be conducive to long-term memory. At the same time, it can also master the basic development technology of the expert system. AI can require role cognition to build a knowledge base composed of production rules by it or further use tool software to develop simple practical expert systems. In order to complete this work, the role cognition needs to formulate development plans, formulate knowledge acquisition strategies, and put them into practice at the beginning, which is a process of continuous deepening. Students must also identify all variables or related factors related to the system, convert these variables and factors into problem solving, and draw corresponding conclusions [19]. After a series of problem solving analysis, role cognition uses production rules to represent knowledge, and the expert system established by this can also be used and experienced by other roles.

Traditional school teaching pays more attention to scores and results and mostly adopts the summative evaluation method of standardized tests. Although the formative evaluation advocated now is also widely promoted by schools, most of them focus on form, and the concept of focusing on scores is still deeply rooted. Although the emergence of AI cannot fundamentally subvert this method of teaching evaluation, it is necessary to use various forms of tests to understand students' mastery of learning content. Teachers not only assume the role of knowledge imparting but also need to have good intellectual literacy and cultivate students' core literacy and moral sentiment. They need to learn to use AI; otherwise, they will be easily eliminated, and they need to reflect on their relationship with AI to enhance their self-worth. In addition, text recognition, speech recognition, image recognition, and biometric recognition can monitor and evaluate the learners' psychological state and attention state in real time according to the learners' words, voices, demeanor, movements, expressions, etc. The visual form presents role cognition in the education system and provides timely feedback for teaching. The AI system can work in a wider range, but the information grasped by each object is relatively shallow, and most of the learners are in a specific cognitive state, lacking personality, emotion and behavior management, family background, learning history, etc.

RETRACTED

The advent of the era of AI has had a huge impact on the traditional perception of teachers' roles, requiring teachers to establish a new outlook on talents, teachers and students, and teaching, and reunderstand the role of teachers. First of all, teachers should establish a new concept of talents that everyone can become a talent, correctly view the differences and individuality of each student, and pay attention to the individualization of students' learning needs [20]. Every student needs to go through good education and guidance to give full play to their potential, create a world of their own, and become useful talents in different fields. Secondly, establish a new concept of teachers and students on the basis of updating the concept of talents. Teachers need to realize that students are independent learners with self-awareness, students are the main body of learning, and students will always be in the dynamic learning process of continuous development. Teachers are the companions, inspirations, and leaders of students' learning. Therefore, teachers and students are two subjects in the same learning activities. This teaching concept highlights the equal participation of teachers and students, joint participation, teaching and learning, and teaching unity.

## 5. Conclusions

Taking the entire education system in Taiyuan City, Shanxi Province, Central China, as an example, this paper uses questionnaire survey method to analyze the effect of AI on role cognition in the education system. The education system targeted by this questionnaire survey involves 8 categories: preschool education, primary education, secondary education, higher education, adult education, computer network education, enterprise education, and social education; the respondents include 368 teachers, 402 students or learners, 118 school managers, and 124 family members of students or learners in all above education categories. The education system can make use of this characteristic or expand on the original basis to meet the needs of students' own learning needs. After all, it cannot replace human learning and innovation. This is the subjective condition for students to form a correct learning attitude and motivation to further enhance their independent learning ability and creativity. From the perspective of technology acceptance, the information literacy of teachers and students is directly related to the perceived ease of use and perceived usefulness of intelligent technology, and such technology perception will largely determine teachers and students' willingness to use intelligent technology and their perceived usefulness. The research results show that the learning of AI courses is strongly dependent on course role cognition, and the construction of role cognition is related to the understanding of course content, teaching methods, and activity methods. Therefore, AI plays a role in role cognition in the education system. The role of the project needs to be systematically analyzed from the aspects of function realization form, resource presentation method, supporting hardware form, teacher-student interaction method, and representation method of works. As a connecter, teachers are limited by the degree of understanding learners, the amount of resources, and data processing capabilities, but the advantage is that they can flexibly monitor and adjust. AI technology is flexible and diverse, it functions in learning and teaching activities in a variety of ways, and there is no agreement on the terminology to describe its role. The results of this paper provide a reference for further researches on the effect of AI on role cognition in the education system.

RETRACTED

## Figures and Tables

**Figure 1:** Effect of AI on role cognition of teachers or couches (a), students or learners (b), school managers (c), and family members (d) in different education categories.

**Figure 2:** Analytical framework of the effect of AI on role cognition in the education system in Taiyuan City.

**Figure 3:** Correlation analysis of AI and role cognition of all 8 (a)–(h) different categories in the education system. (a) Preschool education, (b) primary education, (c) secondary education, (d) high education, (e) adult education, (f)network education, (g) enterprise education, and (h) social education.

**Figure 4:** Analysis of mechanism by which AI affects role cognition in the education system.

**Figure 5:** Factor analysis of AI acting on role cognition of all 8 (a)–(h) different categories in the education system of Taiyuan City. (a) Preschool education, (b) Primary education, (c) secondary education, (d) high education, (e) adult education, (f) network education, (g) enterprise education, and (h) social education.

**Table 1:** Rating system of questionnaire design in the education system of Taiyuan City.

Rating system	Extremely important	Very important	Relatively important	Not very important	Not important
Point	5	4	3	2	1
6 role recognition items					
34 questionnaire questions					
64 descriptions of role cognition of various objects					

**Table 2:** Sampling distribution of each education category in each education system of Taiyuan City.

Education category	Units	Teachers or couches	Students or learners	School managers	Family members
Preschool education	5	43	50	17	17
Primary education	5	51	53	13	15
Secondary education	5	46	44	11	13
High education	5	42	52	19	15
Adult education	5	49	56	16	20
Network education	5	50	48	14	15
Enterprise education	5	46	47	15	15
Social education	5	41	52	13	14
Total	40	368	402	118	124

**Table 3:** Statistics of questionnaire distribution and recovery in each education system of Taiyuan City.

Items	Teachers or couches	Students or learners	School managers	Family members
Questionnaires distributed	368	402	118	124
Questionnaires recovered	348	399	118	113
Recovery rate (%)	94.57	99.25	100	91.13
Valid questionnaires	343	393	117	104
Effectiveness (%)	98.56	98.50	99.15	92.04

**Table 4:** Rating results of effects of AI on different role recognition descriptions in the education system in Taiyuan City (note: PSE: preschool education; PE: primary education; SE: secondary education; HE: high education; AE: adult education; NE: network education; EE: enterprise education; SE: social education).

Role recognition	PSE	PE	SE	HE	AE	NE	EE	SE
Morality	3	5	4	4	5	5	3	2
Discipline	4	3	5	2	4	3	3	3
Knowledge	1	2	3	3	3	5	4	4
Professionalism	3	3	5	5	2	2	5	2
Activities	5	4	3	3	3	4	5	3
Communication	3	1	4	4	4	5	3	4
Guidance	2	3	2	2	2	3	2	4
Consultation	4	5	4	4	3	4	4	5
Research	4	4	2	5	3	4	3	5
Practice	5	5	4	3	4	5	2	3
Goals	3	4	2	4	4	5	4	3
Feedback	4	3	3	2	3	2	3	4

## Data Availability

The data used to support the findings of this study are available from the corresponding authors upon request.
